# Auditory Speech Based Alerting System for Detecting Dummy Number Plate via Video Processing Data sets

**DOI:** 10.1155/2022/4423744

**Published:** 2022-09-02

**Authors:** Meena Deshpande, M. B. Veena, Alachew Wubie Ferede

**Affiliations:** ^1^BMS College of Engineering, Bangalore, Karnataka, India; ^2^Department of Chemical Engineering, College of Biological and Chemical Engineering, Addis Ababa Science and Technology University, Addis Ababa, Ethiopia

## Abstract

Spectrum of applications in computer vision use object detection algorithms driven by the power of AI and ML algorithms. State of art detection models like faster Region based convolutional Neural Network (RCNN), Single Shot Multibox Detector (SSD), and You Only Look Once (YOLO) demonstrated a good performance for object detection, but many failed in detecting small objects. In view of this an improved network structure of YOLOv4 is proposed in this paper. This work presents an algorithm for small object detection trained using real-time high-resolution data for porting it on embedded platforms. License plate recognition, which is a small object in a car image, is considered for detection and an auditory speech signal is generated for detecting fake license plates. The proposed network is improved in the following aspects: Training the classifier by using positive data set formed from the core patterns of an image. Training YOLOv4 by the features obtained by decomposing the image into low frequency and high frequency. The resultant values are processed and demonstrated via a speech alerting signals and messages. This contributes to reducing the computation load and increasing the accuracy. Algorithm was tested on eight real-time video data sets. The results show that our proposed method greatly reduces computing effort while maintaining comparable accuracy. It takes 45 fps to detect one image when the input size is 1280 × 960, which could keep a real-time speed. Proposed algorithm works well in case of tilted, blurred, and occluded license plates. Also, an auditory traffic monitoring system can reduce criminal attacks by detecting suspicious license plates. The proposed algorithm is highly applicable for autonomous driving applications.

## 1. Introduction

Real-time object detection finds its application in autonomous vehicles, manufacturing industries, etc. Limited memory and computation power have made real-time object detection very challenging. Small Objects of interest imply that objects are really small in appearance like mouse, plate jar, bottle or objects are physically large in appearance but still they take up a smaller patch on an image like train, airplane, bicycle, and car [1]. Diversity in input images and its representation makes the job of small object detection complicated. An application for autonomous driving requires end to end detection with less computation time. Even after the success of Deep Neural Network (DNN), there exists a huge difference in performance evaluation metrics (accuracy) of large, small, and medium objects. Two primary approaches of object detection are one-stage approach and two-stage approach. The difference in these approaches is that detection efficiency of one-stage approach is better compared to other approaches. Two-stage approaches which are region-based detectors are low in speed for real-time applications even though they exhibit higher accuracy. Deeper architecture results in higher computation leading to low speed. In practical applications, the major issue is to strike a compromise between speed and accuracy. The evaluation shows that deeper the architecture is the number of layers, which requires higher training parameters. This needs higher resource consumption and larger data to fine tune training parameters. Finally, resulting accuracy is high. But it makes practical application of deeper architecture difficult. For example, faster RCNN can be considered as a baseline model to detect multiscale objects with high performance, but the speed needs to be compromised. Choice of the model is done considering various factors to enhance Mean Average Precision (mAP) like super resolution for obtaining scaling information of small objects, multiscale training [1, 2]. In practical applications like vehicle detection, license plate detection, YOLO is a good choice to consider since it exhibits a good tradeoff between speed and accuracy. There is a significant impact of amount of data on the backbone model. Shallow models work well for scarce data. YOLOv2 offers a simple balance between speed and accuracy. YOLOv2 is ideal for small GPUs, high frame rate videos as it runs at 90 Frames per second (FPS) with mAP comparable to fast R-CNN. But the drawback of YOLOv2 is detecting small objects. Considering all this fact we have chosen YOLOv4 as the backbone model and to reduce the computational load Haar-based training is done. Comparatively low recall and more localization error compared to Faster R_CNN, Struggles to detect close objects because each grid can propose only 2 bounding boxes, and Struggles to detect small objects are the limitations of YOLO.

### 1.1. Context of the Problem with reference to Case Study

In India, the size of the number plate is variable (which may be considered as small objects) and the surveillance purpose CCTV cameras are of low resolution. Hence, automatic number plate recognition remains a challenging problem. This problem of detecting variable size number plate with good accuracy as well as with good speed is addressed in this paper. Organization of the paper is as follows: Section 2 describes the challenges in small object detection; Section 3 briefs related work; Section 4 explains the basics and preliminaries associated with the proposed work; Section 5 introduces the proposed work; Section 6 describes the experimental setup and lists the results followed by conclusion, future work, and references.

Key contributions of this work are shown in Figure 1:

1. YOLOv4 along with Haar cascade training is proposed. In accordance with this low-level and high-level feature information is extracted using Haar cascading. This makes our method practical for real-time object detection (Vehicle and in particular small objects like number plate of the vehicle). The proposed work helps in achieving multiple tasks like small object detection, multiple object detection, reducing computation time, and apparently memory requirement.
2. As a case study for small object detection, license plate detection is studied in this work. License plate forms a small object in the complete image area and detection is achieved using YOLOv4 which is specially designed to overcome the drawback of YOLO and YOLOv2 of localization and small objects detection, respectively, see Figure 1.

## 2. Regarding Small Objects and Detection Challenges

Zhu et al. [1, 3] stated that small objects occupy 20% of an image size. The object is said to be small if the dimensions of bounding box are 20% lower than that of image height and width.

Challenges associated with small object Detection: Small object detection faces several challenges apart from normal object detection like small appearances. Detector gets confused to spot small objects which are of similar appearance and located around.

Also, locating small objects is difficult in the clutter background. Pixels representing small objects are less informative. Furthermore, numbers of available pixels representing the data of small objects are less compared to normal objects. Key features of small objects are eventually lost while going through subsequent DNN. Example, object occupying size of 32 × 32 is represented by one pixel after pooling in VGG16. This makes sliding window, selective search impractical to attain good outputs. Useful data pertaining to small objects with respect to training may get ignored due to widespread use of small objects in the image. This demands to exploit the contents of an image as well as the amount of data significantly impacts the model.

## 3. Related Work

This section reviews work that comprises a deep learning approach to detect small objects and recognize number plates. Expanding Receptive Field YOLO (ERF YOLO) was introduced [4] to optimize YOLOv2 in locating small objects. ERF block was used to expand the receptive field. Low-level information was down sampled by ERF block for obtaining location information and deconvolution was used to up sample the high-level information to obtain feature information. The detection result was obtained by combining these two results. Even though ERF YOLO shows improvement in accuracy the inference time required was high. Two-stage like fast and faster RCNN, and one-stage approaches like YOLOv3 are evaluated for parameters like resource utilization, processing speed along with the backbones like Feature Pyramid Network (FPN), (residual Networks) ResNet, or ResNeXT in [1]. The work clearly states the advantages and disadvantages of the model pertaining to above parameters and changes in these parameters when the size of the object is scaled. This paper provides a detailed comparison of two-stage and one-stage methods. Work concludes that faster RCNN can be considered as a baseline to develop a model from it, but faster RCNN falls short in real-time applications and training is also complex. Hence, YOLO can be good in case of real-time application as even though training time is high, the tradeoff between speed and accuracy is worth applying. Also, the drawback of YOLO is removed in YOLOv2 and YOLOv3. YOLOv2 is not able to detect small objects. Even though YOLOv3 has good accuracy in detecting small objects, speed of YOLOv3 is slow compared to YOLOv2 due to use of DarkNet-53 combined with techniques like skip connections, residual blocks, and up sampling. To overcome this drawback of YOLOv2and YOLOv3, we have used YOLOv4. YOLO-V4 system weight files are small and do not require high hardware requirements. It can also be implemented in PyTorch so that it can be deployed on mobile devices, enabling edge devices to run these models as well, relieving the space constraint of immovable signal capture devices and providing the advantages of high accuracy and high detection rate [5]. Multiple object detection is achieved using YOLOv3 and openCV on KITTI and COCO data sets. The evaluation shows that accuracy obtained for car and heavy vehicles are 95.5% and 96%, respectively, for day images [6]. Work does not show the performance evaluation metrics for real-time data. Also, it is suggested that design can be modified to make the model more robust and suitable for real-time applications. Multiple vehicle tracking is proposed in [7] proposed EYOLO vehicle detection algorithm processing at 35 FPS. The methods involve use of a kalman filter for multiple vehicle tracking. Resource consumption can be reduced by using convolutional neural networks based on the Haar filter. G-Haar-based methods proposed in [8] outperform BNN as G-Haar weight can keep higher computing precision in comparison to binary networks. Local regression tasks using sparse window generation strategy can detect multiscale small objects [9].

Automobile industry related applications like crime tracking, traffic violation tracking gaining fame hence also License plate recognition (LPR). The LPR model is stable and robust due to the use of edge information, texture features, and mathematical morphology. A review on number plate detection and recognition is considered as license plate is a small object in vehicle images. License plate recognition of a Chinese vehicle is proposed in [10] by use of a kernel-based learning machine with deep convolutional features. Main aim was recognition of the Chinese number plate. Abedin et al. [10, 11] proposed license plate recognition but it performed well on only high-quality images. Cloud-based number plate recognition for smart cities was proposed by Polishetty et al. [12] which involves binarization and edge detection, but these approaches are susceptible to complex backgrounds. The merging of CNN and RNN is proposed by Redmon and Farhadi [13] for reading car number plates. The proposed method investigates the blending of RNN and CNN for car number plate detection and recognition. The operational speed of these methods is not clearly mentioned. Also, all these works do not consider real-time scenarios. [14] has addressed the problem of identifying moving vehicles with their number plates. The work involves a database system for identifying the culprit. Most of the works involved used openCV with python. The accuracy of openCV is less than that of YOLOv3 and the speed of detection is less. A real-time vehicle detection and LPR recognition system are presented to address the issue of fake number plates, accuracy, poor quality images, speed, etc. Number plate is detected and recognized from the moving vehicles. [15] proposes YOLOv2 DarkNet based on Alexey's implementation. [16] uses YOLOv2 for fast and accurate license plate detection. Even though the recognition rate achieved was 78.33%, but the results were unsatisfactory for some real-world Automatic License Plate Recognition (ALPR) applications. Author also proposes to explore new CNN architecture to optimize speed.

## 4. Basics and Preliminaries

### 4.1. Basics of YOLO4

YOLO is a real-time object detection model, having three versions, with progressively substantial improvement. YOLOv1 [17] widely known as YOLO is a one-stage network which looks at object detection as a regression problem, hence giving class probabilities and prediction simultaneously for bounding boxes coordinates. Input image is fixed to size by resizing, and later a single convolutional network works on the image. A threshold is put on the resulting detection with the model confidence score On GPU, YOLO detects at a speed of 45 fps. Smaller Fast YOLO achieves the speed of 150 fps. The result is displayed by dividing the input image into a S x S grid of equal width and height of the tensor. Grid cell takes responsibility of detecting objects if the center of the object is inside grid cell. Also, every grid cell is concurrently responsible for predicting confidence scores and bounding boxes presenting the confidence of the model as well as the accuracy of predicting bounding boxes. Background errors in YOLO are less than half as compared to faster RCNN. YOLO struggles in precisely locating small objects. Further, localization error present in YOLO is fixed in YOLOv2 by introducing many new training methods like batch normalization, multi-scale training with input images of higher resolutions, use of default bounding boxes in place of fully connected layers. YOLOv2 focuses on improving localization and recall. This offers a tradeoff between accuracy and speed. Improvements in YOLOv2 allow it to train multi-class data sets like COCO/ImageNet. YOLOv2 fails in detecting small objects because of the resulting low dimensions of the feature map due to input down sampling used for final prediction. These issues of YOLOv2 are addressed in YOLOv3 with remarkable improvements in detecting small objects. YOLOv3 [13, 18] approach developed deeper network consisting of 53 layers termed Darknet53 and it also combines the network with methods like skip connections as in ResNet, residual blocks, and up sampling in order to improve recall precision and Intersection over union (IoU) metrics. Since YOLOv3 consists of 106 layer fully convolutional architecture, it is slow in speed compared to YOLOv2. Low-resolution image performance is improved as YOLOv3 predicts objects at three distinct scales instead of single prediction at last layer. Final detection is done by applying a 1 × 1 kernel on a feature map of three different sizes and three different positions in the network like FPNs. YOLOv3 creates nine anchor boxes and divides them into three areas. Bounding boxes per image are more as each location administers three anchor boxes. Number of boxes predicted by YOLOv3 are 10 times the number predicted by YOLOv2. [19] cost function calculation in YOLOv3 is different from YOLOv4. YOLOv3 uses logistic regression for the bounding box prediction, that is, binary cross entropy loss for each label instead of mean square error for calculating classification loss. Softmax function is not used for class prediction. YOLOv3 obtained a mAP of 37 on the COCO-2017 validation set with input image resolution of 608 × 608, whereas the competing MobileNet-SSD architecture received a mAP of 30. YOLOv4 architecture is used in the current work [20].

Table 1 illustrates the different versions of YOLO [5].

### 4.2. Basics of Haar Cascading

The wavelet transform decomposes the input image into of wavelet images with frequencies namely low-frequency LL containing the source image's vital intelligence, and the high-frequency LH, HL, and HH, which preserve the source image's horizontal, vertical, and diagonal edge details, respectively. Wavelet possesses the ability to localize time-frequency for limited duration. They are adjacent rectangles at distinct positions in an image. Haar-like feature's basis depends on detection of features and encoding the information about the class to be detected. Haar-like features are of three types. The first being edge feature, second is the line feature, and third type is the center-surround feature. Haar feature selection algorithm is based on the foundation of calculating the difference between the sum of black pixels and sum of white pixels. Haar-like features demonstrate fast sum computation by use of integral images. Integral image depends upon the number of pixels in the rectangle. Since it does not depend on individual pixel computation speed is high. As it is based on the fundamental of Haar wavelet, it is called Haar-like. Integral image consists of small units, representing a given image.

The integral image is described as

(1) $$\begin{array}{c} ii\left(x,y\right)\;=\sum_{x^{\prime }\leq x,y^{\prime }\leq y}i\left(x^{\prime },y^{\prime }\right), \end{array}$$

where *ii*(*x*, *y*) is the integral image and *ii*(*x*′,  *y*′) is the original image.

Haar Cascade Classifier is a method utilized for detecting objects [21–23]. It has four points for object detection, such as Haar-like features, integral image, AdaBoost learning, and Cascade Classifier. Advantage of integral image is its capability of performing basic operations in a very less processing time. Use of integral image made cascade classifier to run in real time.

### 4.3. Speech Alerting Unit

The speech alerting system is to assure the redundancy mapping and signal strength orientation of overall data under the processing channel. As the authors discuss a detailed signal analysis via a speech alerting in [24] the orientation assures the process is dependent on mapping and extraction of results via a spoken grammar library or lookup database systems. The similar pattern of signal compression is discussed in [25] with an order of ration inter-dimensional signal processing. The fall detection based alerting system discussed in [26] for feature-based discussion support. In the proposed system architecture, the behavioral model assures the processing and detection of dummy name plates via a video data sets through an approach of interdependent decision support of alert management.

## 5. Proposed Work

The proposed work helps in achieving multiple tasks like small object detection, multiple object detection, reducing computation time, and apparently memory requirement. As a case study for small object detection, license plate detection is studied in this work. Proposed approach consists of diverse layers like pre-processing, feature extraction, training, testing, vehicle license plate detection layer, and TTS conversion. A training set is generated containing a huge amount of positive and negative data for automatic detection and recognition of license plates in a real-time video during the pre-processing stage. Positive images are obtained by cropping core sub-image with the aspect ratio same as that of license plate by use of positive training data set computation time is further reduced. Pre-processing is followed by feature extraction. Feature extraction includes extracting features like length, width-height of the object. Haar features were extracted and trained using Haar cascading [27]. The Haar cascade classifier was trained on a batch of positive and negative samples which were sewed up later together to form a vector file to generate an xml file. In addition, use of GPU (Graphics Processing Unit) increased the computation speed and processes at 45 frames per second. Purpose of using Haar is twofold. Haar cascading reduces the computation and memory requirement as well. Testing phase is executed after training phases which checks whether the detected object is correct or incorrect. YOLOv4 predicts moving object detection using CSPDarknet53 frameworks. YOLOv4 is used to predict the bounding box and to calculate the confidence score of predicted vehicles using a single convolutional neural network. Input image is split in to *S* × *S* grid. *m* bounding boxes are produced inside each grid. The bounding box with probability of class greater than threshold represents detected object.

Speech synthesis (or Text to Speech) is the computer-generated simulation of human speech. It converts human language text into human-like speech audio. In this tutorial, you will learn how you can convert text to speech in Python [28]. Text-to-speech reads words on webpages, smartphones, etc., and converts written text to a phonemic representation (Sounds of a word), further it converts the phonemic representation to waveforms using WaveNet that can be output as sound. The block diagram below represents the working of the same. TTS is built using python [29]. Python facilitates with different APIs to convert text to speech. We have used gTTS API which enables us to read text on-screen supporting different languages like Kannada, Tamil, English, and Hindi [30].

The Algorithm 1 operates on a folder which contains image files.

## 6. Experimental Setup

### 6.1. Hardware Requirements and Annotation

Proposed method is verified by carrying out experiments on the data collected by real-time cameras. Camera used is SC-IS42BP-I (*Z*) (*S*) (*W*). Key features of the camera is 1/2.7 MP progressive scan CMOS. Max resolution of the camera is 2688 × 1520 @1–25fps. It supports low bit-rate, low delay, and ROI enhance coding Quad Stream support. Images were collected by using high-definition camera with 2688 × 1520 resolutions. Cameras used reflected real-time scenario of the traffic for 24 hours in variable traffic scene. Data set is split as 40% for training, 40% for testing, and 20% for validation, in accordance with the division protocol proposed by Tanwir [31] in the SSIG data set. We have used LabelImg annotation tool, a graphical annotation tool to graphically label images. It is coded in Python, and the graphical interface is provided by QT. Annotation is saved as xml file in YOLO format. This study focuses on various parameters such as the x-coordinate of the bottom-left corner of the rectangle (*x*), the y-coordinate of the bottom-left corner of the rectangle (*y*), the width of the rectangle (*w*), and the height of the rectangle (*h*). According to research, low-level layers carry location information and high-level layers consist of information pertaining to features [32]. To gauge the performance of the proposed algorithm, 2424 images were used. Some types of License plates appeared more than other, since vehicle images are collected from real-traffic scenes. Real-time data collection made data set challenging due to variation in illumination, background, plate color, font, etc. For creating positive training set images were cropped to the core sub-image with same aspect ratio as that of license plate [33]. This increases the detection rate of license plates. Class IDs like 0, 1, 2, 3, 4 are provided for detection of yellow, white, black, green, red colored number plates. This is demonstrated in Table 2. Example: <Class ID> <*x*><*y*><*w*><*h*> Example of annotation.

### 6.2. Software Requirements

Tensorflow and OpenCV [4] have been of great aid in providing cross-platform support for the execution of numerous vision algorithms, making analysis easier. Tensorflow and OpenCV are used for configuring the resource-constrained setting. The proposed method is implemented on Python v3.8 on a PC with 3.4 GHz i7 quad core CPU using C++. All experiments were conducted by using Anaconda Navigator 2.0, Pandas v1.0.5, Open-source API–Keras v2.2.0, Backend framework used is–Tensorflow-gpu v2.2.0, Intel Core i7 9th generation processor (16 GB RAM) using Windows 10, NVIDIA GeForce RTX 1080Ti GPU [34].

### 6.3. Experimental Test Observations

Proposed algorithm detects multiple vehicles, and license plates are detected with different color number plates.

GUI entry table consists of an alert entry which has same columns namely filename, LPR result, and the confidence with which it predicts. The algorithm checks for specific conditions. If conditions are not satisfied, then the data pertaining to that number plate are logged in alert table. Conditions are that the confidence score should be higher than 40% and the number of characters predicted should be between 8 and 10.

File No. Filename, LPR result, and the Confidence score is detected.

Figure 2 represents the vehicle detection of real-time data sets with LPR number, color, and the efficiency of detection.  Figure 3 proposed block diagram of auditory Speech based alert system for detecting fake number plates.  Figure 4 illustrates Text to speech conversion using python [28]. This work can detect the number plates which are blurring and tilted.  Figure 5 illustrates architecture of YOLOv4.  Figure 6 shows Annotation of Car license plate.  Figure 7 shows the proposed method of real-time video indicating the detected vehicle with license plate.  Figure 8 illustrates license plates at different angles.

Table 3 shows the result of LPR detection with confidence score. It can also be observed that multiple vehicles in an image are also detected.

The algorithm is subjected to real-time videos containing vehicles of variable sizes for speed analysis. In comparison to the YOLOv3 approach, there is 3 percent gain in speed [35]. Average accuracy, precision recall values obtained for six different real-time videos captured at real time are tabulated in Table 4. Accuracy is 97% improved by 3.2% greater accuracy than existing YOLOv3.

Three metrics are considered for evaluating object detection algorithm performance, namely accuracy, precision, and recall. Table 4 gives the performance metrics for the proposed algorithm.

Proposed algorithm is able to detect LPR at different angles, different fonts, and colors.

Alert messages generated from LPR data in GUI are conveyed to traffic in charge from dashboard and accordingly an enquiry is done for false number plate.  Table 5 demonstrates the performance estimation and speech alert management of incoming patterns.  Table 5 also computes the inter-dependency of information signal processing and response time computation for particular signal and speech cum alerting message. The process assure the computational statistics of computation with reference to signal strength and processing delay.

## 7. Conclusion and Future Work

In this paper, we proposed modified YOLOv4 with Haar cascading based feature extraction and training for detecting small objects like License plates. OpenCV along with python was used for character segmentation and recognition. With the proposed algorithm, we were able to reduce the memory consumption and computation time. Haar CNN was used to train the model. This approach processes images with a frame rate of 45 (fps) which is greater than YOLOv3. Results on the real-time data captured by camera shows the operational compression of the model still achieving mAP of 87%. Proposed algorithm can significantly improve the camera-based License plate detection system for autonomous driving, and can contribute remarkably in the applications of autonomous driving. In future work, different wavelets like contourlets can be used for extracting features. Also, the network structure can be improved further. Researchers can also focus on a combination of feature extractors like GLCM and Haar to improve real-time performance as well as accuracy. The proposed system computes with a speech based alerting system and estimated performance of 97.23% with reference to selection of alerting message and information selection. The framework assures the detection and processing of dummy plates via video processing data sets. Recently, objects on dark, low-resolution, blurry images and tough angles, all vehicle types are implemented. Future work can be improving the detection of Decodes license plate, vehicle type (e.g., SUV, van, pickup truck), vehicle make model (e.g., Honda Accord), color, and orientation which Ignores bumper stickers, car signs, etc.

## Figures and Tables

**Figure 1:** Objects having a big appearance but occupying a small portion of the image like a car and bike. The license plate at different angles and with poor visibility.

**Figure 2:** Functional diagram of proposed auditory alert system for detecting fake number plates.

**Figure 3:** Proposed block diagram of auditory speech based alert system for detecting fake number plates.

**Figure 4:** Text to speech conversion using python [28].

**Figure 5:** Architecture of YOLOv4.

**Figure 6:** Annotation of car license plate.

**Figure 7:** GUI of the proposed method of real-time video indicating the detected vehicle with license plate.

**Figure 8:** Figure illustrates license plate at different angles, blurred, and occluded circumstances.

**Algorithm 1:** Object detection using YOLOv4 with Haar based training.

**Table 1:** Comparison of different versions of YOLO [5].

YOLO v3	YOLO v2	YOLO	Detector
	—	—	Proposal

Darknet	Darknet	GoogleNet	Backbone

Variable	Fixed	Fixed	Input image
	<50	<25 VGG	Speed

CVPR18	CVPR17	CVPR16	Published in

Sigmoid instead of a softmax	SGD	SGD	Optimization

Cross-entropy error terms + bounding box regression + object confidence (object confidence and class predictions in YOLO v3 are predicted through logistic)	Class sum square error loss + bounding box regression + object confidence + background confidence	Class sum square error loss + bounding box regression + object confidence + background confidence	Loss function
	Yes	Yes	End-to-end train

C and python	C	C	Language

Darknet-53	Darknet-19	Darknet	Deep learning platform

Achieves good performance for small objects as well as with more speed	Achieve high accuracy and high speed propose a faster darknet 19; improved the speed and accuracy by using several existing strategies; YOLO 9000 can detect over 9000 object categories in real-time limitations: struggling in detecting small objects	First unified detector framework (elegant and efficient) exclude RP method completely, faster than previously proposed detectors. YOLO and fast YOLO run at 45 and 155 FPS, respectively limitations: have difficulty to localize tiny objects. Dramatics accuracy falls as compared to the state of art	Merits and limitations

**Table 2:** Table represents class ID for different colors of number plate.

Sl. no.	Class	Class ID
1	Yellow plate	0
2	White plate	1
3	Black plate	2
4	Green plate	3
5	Red plate	4

**Table 3:** Output file indicating the number on license plate with the confidence score.

Sl. no	Name of the file	Detected license plate result	Confidence score
1	192.168.0.141_1568622026.png	KA04ML4979	99.3%
2	192.168.0.141_1568622052.png	KA03NN5197	98.0%
3	192.168.0.141_1568622061.png	KA05MU4437	98.1%
4	192.168.0.141_1568622244.png	KA04AB8892	99.4%
5	192.168.0.141_1568622192.png	HR26BP2529_M0AKH_,	99.4%_70.0%
6	192.168.0.141_1568622192.png	HR26BP2529_M0AKH_,	99.4%_70.0%
7	192.168.0.141_1568622240.png	AAO5AF881_KA019661_,	79.8%_82.6%
8	192.168.0.141_1568622111.png	KA51AC6318_A15I1K_,	99.3%_72.0%
9	192.168.0.141_1568621965.png	KA01AE0014_B191_,	98.5%_42.1%

**Table 4:** Table indicates the values of different evaluation metrics like average accuracy, precision, recall tested on six different real-time videos.

Video	Average accuracy	Precision	Recall
1	98	0.8	0.73
2	96	0.89	0.72
3	99	0.89	0.73
4	98	0.82	0.72
5	82	0.79	0.8
6	88	0.8	0.72

**Table 5:** Speech signal alerting and management tabulation and performance estimation.

Sample name	Speech signal strength (Hz)	Processing delay (sec)	Response time (sec)	Alerting subject accuracy (%)
192.168.0.141_1568621723.png	147	0.36	0.025	97.21
192.168.0.141_1568621724.png	125	0.37	0.231	98.21
192.168.0.141_1568621798.png	126	0.36	0.321	97.11
192.168.0.141_1568621843.png	175	0.36	0.211	97.34
192.168.0.141_1568621897.png	123	0.36	0.231	96.98
192.168.0.141_1568621904.png	164	0.36	0.112	97.11
192.168.0.141_1568622026.png	128	0.36	0.921	95.21
192.168.0.141_1568622052.png	197	0.36	0.143	97.84
192.168.0.141_1568622061.png	201	0.36	0.021	98.21
192.168.0.141_1568622244.png	122	0.36	0.045	92.12
192.168.0.141_1568622192.png	153	0.37	0.134	97.12
192.168.0.141_1568622192.png	185	0.37	0.043	98.02
192.168.0.141_1568622240.png	142	0.36	0.082	98.21
192.168.0.141_1568622111.png	123	0.36	0.214	97.12
192.168.0.141_1568621965.png	163	0.36	0.728	97.21

## Data Availability

The data sets used and/or analyzed during the current study are available from the corresponding author on reasonable request.
